# Comprehensive Comparison of Three Different Immunosuppressive Regimens for Liver Transplant Patients with Hepatocellular Carcinoma: Steroid-Free Immunosuppression, Induction Immunosuppression and Standard Immunosuppression

**DOI:** 10.1371/journal.pone.0120939

**Published:** 2015-03-27

**Authors:** Yuan-Yuan Liu, Chang-Ping Li, Ming-Sheng Huai, Xiao-Meng Fu, Zhuang Cui, Lin-Lin Fan, Shu Zhang, Yuan Liu, Jun Ma, Guang Li, Zhong-Yang Shen

**Affiliations:** 1 Department of Health Statistics, School of Public Health, Tianjin Medical University, 22 Qi-Xiang-Tai Road, Heping District, Tianjin, 300070, China; 2 Department of Transplantation, Tianjin First Center Hospital, 24 Fu-Kang Road, Nankai District, Tianjin, 300192, China; 3 Follow-up Center, Department of Transplantation, Tianjin First Center Hospital, 24 Fu-Kang Road, Nankai District, Tianjin, 300192, China; 4 Department of Biology, School of Basic Medical, Tianjin Medical University, 22 Qi-Xiang-Tai Road, Heping District, Tianjin, 300070, China; Penn State University, UNITED STATES

## Abstract

The different choices of immunosuppression (IS) regimens influenced the outcomes of liver transplantation. Steroid was applied as a standard IS to prevent and treat rejections. However, steroid-related complications were increasingly prominent. This study compared the efficacy and safety of standard IS regimens with the efficacy and safety of steroid-free IS regimen and induction IS regimen in Chinese liver transplantation recipients for hepatocellular carcinoma (HCC). A total of 329 patients who underwent liver transplantation from January 2008 to December 2012 were retrospectively reviewed. Three different groups of patients received standard triple-drug IS regimen of steroid, tacrolimus (TAC) and mycophenolate mofetil (MMF) (triple-drug regimen group; *n*=57), induction-contained IS regimen of basiliximab, steroid, TAC and MMF (BS group; *n*=241), and induction-contained and steroid-free regimen of basiliximab, TAC and MMF (SF group; *n*=31), respectively. There were no significant differences in terms of patient, tumor-free and graft survival rates. The acute rejection rate and rejection time were equivalent in different groups. But compared with BS group, higher incidences of biliary complications (11.52% vs. 30.77%, *p*=0.013) and graft dysfunction (0.48% vs. 13.64%, *p*=0.003) were observed in SF group. Furthermore, compared with the two groups, incidence of pleural effusion was also higher in SF group (15.79%, 11.96% vs. 45.45%, respectively, both *p*<0.01). And a trend towards less proportion of *De novo* diabetes was revealed in SF group. Although it was found that patient, tumor-free and graft survival rates were equivalent among three IS regimens, higher incidences of complications were demonstrated in steroid-free regimen in patients for HCC. These findings suggested that steroid-free IS regimen has no clear advantages in comparison with standard IS regimens for liver transplant recipients with HCC and the postoperative complications should be treated with concentrated attention.

## Introduction

As a common malignancy worldwide, the incidence and mortality of hepatocellular carcinoma (HCC) varies widely with geographical region. Viral infection, mainly in chronic hepatitis B virus (HBV) and/or hepatitis C virus (HCV) infection, is the predominate cause of HCC globally [1]. Epidemiological studies have established the linkage between HBV infection and HCC. The results indicate that due to the endemic feature of long-term chronic HBV infection, HCC is more prevalent in Asia [2] especially in China. About 55% of newly diagnosed HCC cases [3, 4] all over the world are from China and the similar status is observed in cancer dead cases [5].

Orthotopic liver transplantation (OLT) is proved to be an efficient treatment to extend life for HCC patients with hepatitis virus infected. Immunosuppression (IS) plays an indispensable role in overall process before and after OLT. The usage of IS reduces the acute and chronic rejections, which are the severe side effects after transplantation. Meanwhile the wide usage of IS brings some side effects. Evidences indicated that quit a few of the long-term complications of liver transplantation (LTx) were caused by IS side effects rather than chronic rejection, and in other words transplant recipients were being overimmunosuppressed [6]. Thus immunosuppressive regimens were explored cautiously in order to balance the reduction of rejections and avoidance of side effects [7–9]. The different choices of immunosuppressive regimens were critical for the outcomes after LTx. Since the triple-drug regimen of azathioprine (AZA), prednisone and antilymphoid globulin was introduced to the field of LTx in 1968 [10], the change of the regimens had brought the increase of patient, graft and disease-free survival rates. Up to 1980s, two revolutionized IS, Cyclosporine (CsA) and Tacrolimus (TAC), were applied as the pivotal drugs in LTx. The former was reported crucially to reduce the incidence of allograft rejection combining with corticosteroids (CS) and AZA. The latter was reported with fewer steroid-resistant rejection episodes in a landmark study which was developed in the United States (US) in 1994 [11]. Till now, standard regimen of steroid and calcineurin inhibitors (CNIs) is the most extensively treatment which is applied in the world.

Nowadays, researches are carried out to attempt CS avoidance or early withdrawal for the aim of reducing corticosteroid-related adverse effects, such as diabetes mellitus, hypertension, osteoporosis, fractures and serious infections [12–14]. Therefore, induction therapy has been used to avoid steroid use or delay CNIs use in the preoperative period with the effect of preventing acute rejection. And the proportion of recipients who receive induction therapy has increased from approximately 20% [15] to 30% in the US till 2011. The same situation exists in other countries over the world since 2000 [16]. Basiliximab, an anti-interleukin-2 receptor monoclonal antibody (IL2-RA), is used more commonly in LTx as induction IS in China.

Compared with the convincing proofs of the benefits of induction in acute rejection and graft survival [17, 18] in kidney transplantation, researches are insufficient in LTx. Specially, the IS regimen without steroid was applied originally in western LTx recipients with HCV infection. In the early stage of the aforementioned regimen, the fewer cases were used in LTx recipients for HCC. Recently, the IS therapy without steroid was applied in HCC recipients, and meanwhile the induction IS therapy sprung up. Although several researches had evaluated the effectiveness of IS therapy for HCC recipients with or without steroid [19–21], the grouping was simple and the induction IS therapy was not studied systematically. In this study, the grouping was elaborated, and the research was systematical. This study carried out not only the comparison of the IS therapy with or without steroid but also the difference between the induction IS therapy and the standard IS therapy, using the data from the same origin of China.

## Materials and Methods

### Ethics Statement

This study was approved by the Ethics Committee of Tianjin First Center Hospital and confirmed to the ethical guidelines of the Declaration of Helsinki. None of the transplant donors were from a vulnerable population and all donors gave their consent freely.

### Study Population

This study was a retrospective review of recipients and donors who underwent LTx at Oriental Organ Transplant Center of Tianjin First Center Hospital between January 2008 and December 2012. All patients were followed-up until December 2013. In addition, the data of LTx recipients in Oriental Organ Transplant Center of Tianjin First Center Hospital had good representative in China, and one third of Chinese LTx recipients accepted operation of LTx in this center.

Patients who were pediatric liver transplantation patients (age <18 years), had undergone retransplantation, multiple organ transplantation, liver transplantation for acute/fulminant liver failure, and ABO-incompatible liver transplantation were excluded. Patients were also excluded if they had antoimmune hepatitis.

Patients with symptomatic HCC, HCC recurrence after primary liver resection or pre-transplant HCC patients without symptoms were all included. 319 of these patients underwent liver transplantation due to the presence of a HCC on a cirrhotic liver. The cause of the underlying liver disease in these patients included HBV infection in 257, HCV infection in 52, HBV-HCV co-infection in 10. 6 patients underwent liver transplantation because of the presence of a HCC without a cirrhotic liver. HBV was the reason of underlying liver disease for these 6 patients. In addition, 4 patients had HCC, and it was found at pathologic examination of the liver transplanted for a chronic liver disease (so-called incidental tumors). The cause of the liver disease in these patients was HBV infection.

### Immunosuppression Regimens

Patients who were in the triple regimen group (*n* = 57) received methylprednisolone in combination with TAC and mycophenolate mofetil (MMF). Patients who were in the steroid-free (SF) group (*n* = 31) received basiliximab, TAC with or without MMF. In the SF group, MMF was used for 74.19% (*n* = 23) of the subjects, and 25.81% (*n* = 8) of the subjects only received basiliximab and TAC. In the basiliximab with steroid (BS) group (*n* = 241), methylprednisolone was used. In group of BS, 220 (91.29%) recipients received basiliximab, methylprednisolone and TAC plus MMF, and MMF was not used for 21 (8.71%) recipients.

Methylprednisolone was administered as an intravenous dose of 500 mg ~ 1000 mg during the transplantation process, and TAC was administered as an oral dose of 0.10 to 0.20 mg/kg/day to achieve the whole blood trough concentration in the range of 8 to 10 ng/ml in 1 month postoperative, and the levels were maintained at 5 to 8 ng/ml during the first 3 months and at 5 ng/ml afterwards.

In BS group and SF group, 20 mg intravenous basiliximab was administered during the transplantation process, and the same dose was syringed on the fourth day postoperatively.

100 mg/day of intravenous methylprednisolone was administered for patients in the triple regimen and BS groups from the first day postoperative to the fourth day. From the fifth day postoperative, 20 mg/day of oral methylprednisolone was administered for patients and a gradual tapering schedule was followed to discontinue after 30 days postoperative.

MMF was administered at the dose of 750 mg twice per day, and it was also discontinued after a gradual tapering schedule until half a year postoperative.

All acute rejection episodes were confirmed by liver biopsy based on the Banff criteria [22] before antirejection treatment. If the rejection was mild to moderate, the dose of tacrolimus was increased. If the rejection was severe, patients were given 500 mg methylprednisolone for 3 days.

Recurrence of HCC was monitored by postoperative alpha-fetoprotein level and confirmed by computed tomography (CT).

### Infection and Prophylaxis

Antiviral prophylaxis for hepatitis recurrence mainly included lamivudine, entecavir, adefovir and telbivudine for combination therapy or monotherapy.

Cytomegalovirus (CMV) infections were monitored by protein pp65 with the immunofluorescence test before transplantation, and subsequently on 2, 4, 6, 8, 10, and 12 weeks post-transplantation.

### Study Assessments

The primary endpoints were patient overall survival (OS), graft survival and tumor-free survival. The secondary endpoints were acute rejection rate and incidence of complications.

### Statistical Analysis

Continuous variables were reported as mean and standard deviation or median and inter-quartile range (IQR) according to the distributions of variables. Categorical variables were expressed as frequencies and percentages. Kruskal-Wallis H test, chi square test or Fisher test were applied for univariate analysis. Life-tables and Kaplan-Meier analysis with log-rank test were used for OS, graft and tumor-free survival analysis between different IS groups and survival curves were provided respectively. Cox proportional hazards regression analysis was conducted for univariate and multivariate survival analysis to identify the predictors of survival. Crude and adjusted hazard ratios (HRs) with 95% confidence interval (CIs) were reported. All statistical test with 2-tailed P<0.05 indicated statistical significance. And the statistical analyses were all performed by SPSS 16.0 (SPSS Inc, Chicago, IL, USA).

## Results

### Preoperative Clinical Characteristics of Recipients

Of the 1163 recipients who received a liver transplantation at Oriental Organ Transplant Center of Tianjin First Center Hospital, 329 were eligible for this study between January 2008 and December 2012 (Fig. 1). Recipients were divided into 3 groups, which were triple regimen group (*n* = 57), BS group (*n* = 241) and SF group (*n* = 31). Median follow-up time was 18.00 (3.32, 40.58) months for all recipients, and for triple regimen group, BS group and SF group was 34.30 (11.17, 53.60), 17.17 (1.33, 38.13), 10.47 (1.00, 26.07), respectively (*p*<0.001). Above all, 300 (91.19%) recipients were male while only 29 (8.81%) were female. And the mean age of recipients were 52.69 ± 9.12 years with a concentrated range of 50 to 64 years. None of them had CMV infection. The distribution of HBV infection, HBV and HCV co-infection were significantly different in the three groups (Table 1). In comparison with BS group, the incidence of HBV infection was lower in SF group (*p* = 0.012).

**Fig 1:** Flow chart of patients selection.

**Table 1:** Preoperative clinical characteristics of recipients of three IS regimens.

Characteristic	Triple (*n* = 57)	BS (*n* = 241)	SF (*n* = 31)	*P*-value
Gender				
Male	54 (94.74)	218 (90.46)	28 (90.32)	0.719
Female	3 (5.26)	23 (9.54)	3 (9.68)	
Age (years)				
18~	0 (0.00)	6 (2.49)	0 (0.00)	0.686
35~	24 (42.11)	79 (32.78)	11 (35.48)	
50~	28 (49.12)	129 (53.53)	17 (54.84)	
65~	5 (8.77)	27 (11.20)	3 (9.68)	
BMI^§^				
<18.5	1 (1.75)	6 (2.51)	0 (0.00)	0.681
18.5~	33 (57.89)	134 (56.07)	16 (51.61)	
25~	23 (40.35)	99 (41.42)	15 (48.39)	
Child-Pugh score				
A	24 (42.11)	109 (45.23)	13 (41.94)	0.614
B	18 (31.58)	91 (37.76)	14 (45.16)	
C	15 (26.32)	41 (17.01)	4 (12.90)	
MELD score				
6~	19 (33.33)	89 (36.93)	14 (45.16)	0.601
10~	30 (53.63)	128 (53.11)	13 (41.94)	
20~	7 (12.28)	18 (7.47)	4 (12.90)	
30~	1 (1.75)	6 (2.49)	0 (0.00)	
HBV positive	46 (80.70)	195 (80.91)	19 (61.29)^a^	0.039
HCV positive	12 (21.05)	37 (15.35)	9 (29.03)	0.129
HBV and HCV co-infection^¶^	4 (7.14)	4 (1.78)	2 (8.00)	0.027
Cirrhosis	57 (100.00)	237 (98.34)	29 (93.55)	0.126
Preoperative diabetes mellitus	8 (14.04)	49 (20.33)	6 (19.35)	0.554
Preoperative hypertension	4 (7.02)	38 (15.77)	8 (25.81)	0.057
Downstaging				
Systemic chemotherapy only	0 (0.00)	2 (0.83)	0 (0.00)	0.143
RFA only	4 (7.02)	32 (13.28)	4 (12.90)	
TACE only	20 (35.09)	67 (27.80)	6 (19.35)	
PEI only	0 (0.00)	0 (0.00)	0 (0.00)	
Combination therapy	4 (7.02)	49 (20.33)	5 (16.13)	
None of the therapy above	29 (50.88)	91 (37.76)	16 (51.61)	
TNM staging^★^				0.288
Stage I	3 (5.36)	24 (10.17)	1 (3.33)	
Stage II	4 (7.14)	18 (7.63)	2 (6.67)	
Stage IIIA	3 (5.36)	5 (2.12)	4 (13.33)	
Stage IIIB	41 (73.21)	166 (70.34)	20 (66.67)	
Stage IIIC	0 (0.00)	5 (2.12)	0 (0.00)	
Stage IV	5 (8.93)	18 (7.63)	3 (10.00)	
Vascular invasion	22 (38.60)	80 (33.20)	17 (54.84)	0.056
Milan criteria	22 (38.60)	75 (31.12)	5 (16.13)	0.093
Preoperative antiviral therapy	38 (66.67)	155 (64.32)	14 (45.16)	0.094
Preoperative AFP level, ng/ml^※^	63.06 (10.50, 663.10)	29.78 (5.48, 456.02)	32.24 (8.75, 387.10)	0.389
Number of tumors^♦^	2 (1, 4)	2 (1, 4)	2 (1, 6)	0.955
Diameter of largest tumor, cm^▲^	3.50 (2.08, 6.88)	4.00 (2.50, 7.00)	5.50 (3.38, 10.25)	0.052
Sum of tumor diameters, cm^☯^	6.10 (3.00, 10.62)	5.80 (3.20, 10.00)	10.00 (5.25, 11.75)	0.126

Categorical variables were expressed as number (percentage) while continuous variables were reported as median (IQR).

BMI: body mass index; MELD: model for end-stage liver disease; HBV: chronic hepatitis B virus; HCV: hepatitis C virus; RFA: radiofrequency ablation; TACE: transarterial chemoembolization; PEI: percutaneous ethanol injection; AFP: alpha-fetoprotein.

^§^ 2 cases reported with missing BMI in group BS were deleted;

^¶^ 1 case in triple regimen group, 16 cases in group BS and 6 cases in group SF reported with missing data were deleted;

^★^1 case in triple regimen group, 5 cases in group BS and 1 case in group SF reported with missing data were deleted;

^※^ 1 case in triple regimen group, 1 case in group BS reported with missing data were deleted;

^♦^ 1 case in triple regimen group, 18 cases in group BS and 3 cases in group SF reported with missing data were deleted;

^▲^ 1 case in triple regimen group, 7 cases in group BS and 1 case in group SF reported with missing data were deleted;

^☯^ 3 cases in triple regimen group, 30 cases in group BS and 6 cases in group SF reported with missing data were deleted.

^a^ *p* = 0.012 for comparison with group BS.

According to the 6^th^ edition UICC TNM classification of HCC (2002), of all recipients, 28 (8.51%) recipients were stage I; 24 (7.29%), stage II; 12 (3.65%), stage IIIA; 227 (69.00%), stage IIIB; 5 (1.52%), stage IIIC; 26 (7.90%), stage IV; and 7 (2.13%) unknown due to insufficient pathological data.

However, no significant difference was observed in the distribution of gender, age, BMI, Child-Pugh score, MELD score, TNM staging and other categories. No significances of preoperative AFP level, number of tumors, diameter of largest tumor and sum of tumor diameters were reported, either. Among the downstaging treatments, TACE monotherapy was the most common one in three groups, and then combination therapy was followed.

### Postoperative Complications

Table 2 showed the postoperative complications of the recipients of three IS groups. No significant differences were revealed in some of the postoperative complications, including the incidence of infection, renal failure, vascular complications, intra-abdominal complications, pulmonary edema, PTLD, GVHR, chronic rejection, HBV recurrence, *De novo* diabetes and *De novo* hypertension. Nevertheless, compared with BS group, a higher proportion of recipients experienced biliary complications and graft dysfunction (*p* = 0.013, 0.003, respectively) in SF group. Furthermore, recipients in SF group also suffered a higher incidence of pleural effusion than the other two groups (*p* = 0.006, <0.001, respectively). Besides, recipients in triple regimen group showed a higher incidence of CMVpp65 antigenemia compared with BS group (*p* = 0.001).

**Table 2:** Postoperative complications of recipients of three IS regimens.

Postoperative complications	Triple	BS	SF	*P*-value
Postoperative infections ^§^ ^☯^	11 (19.30)	32 (14.75)	5 (19.23)	0.632
Biliary complications ^¶^ ^☯^	13 (22.81)	25 (11.52)	8 (30.77) ^a^	0.008
Renal failure ^▲^	2 (3.51)	7 (3.35)	3 (13.64)	0.076
Graft dysfunctions ^★^ ^▲^	1 (1.75)	1 (0.48)	3 (13.64) ^b^	0.003
Vascular complications ^※^ ^☯^	3 (5.26)	5 (2.30)	2 (7.69)	0.130
Intra-abdominal complications ^♦^ ^▲^	9 (15.79)	31 (14.83)	6 (27.27)	0.317
Pleural effusion ^▲^	9 (15.79)	25 (11.96)	10 (45.45) ^c^	<0.001
Pulmonary edema ^▲^	0 (0.00)	1 (0.48)	1 (4.55)	0.186
CMVpp65 antigenemia ^☯^	6 (10.53)	2 (0.92) ^d^	2 (7.69)	0.001
PTLD ^■^	0 (0.00)	1 (0.55)	0 (0.00)	1.000
GVHR ^■^	0 (0.00)	2 (1.10)	0 (0.00)	1.000
Chronic rejection ^■^	1 (1.75)	2 (1.10)	0 (0.00)	0.655
HBV recurrence ^♠^	3 (6.12)	8 (3.64)	1 (3.70)	0.684
*De novo* diabetes ^◇^	14 (28.57)	32 (18.29)	3 (14.29)	0.223
*De novo* hypertension ^○^	6 (11.32)	13 (7.03)	2 (9.52)	0.587

CMV: cytomegalovirus; PTLD: post-transplant lymphoproliferative disorder; GVHR: graft-versushost reaction; HBV: chronic hepatitis B virus.

^§^ Postoperative infections included pulmonary infection, catheter-related sepsis, urinary tract infection, wound infection and opportunistic infection;

^¶^ Biliary complications included anastomotic biliary strictures, intrahepatic biliary strictures and bile leakage;

^★^ Graft dysfunctions included primary graft non-function and delayed graft function;

^※^ Vascular complications included hepatic artery embolism, portal vein embolism, hepatic vein/inferior vena cava stenosis/embolism and portal vein stenosis/pylethrombosis;

^♦^ Intra-abdominal complications included intra-abdominal bleeding and intra-abdominal collection/abscess.

^▲^ 32 cases in group BS and 9 cases in group SF reported with missing data were deleted;

^☯^ 24 cases in group BS and 5 cases in group SF reported with missing data were deleted;

^■^ 59 cases in group BS and 11 cases in group SF reported with missing data were deleted;

^♠^ 8 cases in triple regimen group, 21 cases in group BS and 4 cases in group SF reported with missing data were deleted;

^◇^ 8 cases in triple regimen group, 66 cases in group BS and 10 cases in group SF reported with missing data were deleted;

^○^ 4 cases in triple regimen group, 56 cases in group BS and 10 cases in group SF reported with missing data were deleted.

^a^ *p* = 0.013 for comparison with group BS.

^b^ *p* = 0.003 for comparison with group BS.

^c^ *p*<0.001 for comparison with group BS; *p* = 0.006 for comparison with Triple-drug group.

^d^ *p* = 0.001 for comparison with Triple-drug group.

### Acute Rejection

During the study period, a total of 19 recipients experienced biopsy-proven acute rejection. The characteristics of recipients who suffered acute rejection were summarized in Table 3. There were 3 (5.26%) recipients occurred in the triple regimen group, 14 (5.81%) recipients and 2 (6.45%) recipients were in BS group and SF group, respectively. And the incidences of acute rejection were equivalent for the three IS regimen groups (*p* = 0.926) as well as the rejection time (*p* = 0.861).

**Table 3:** Acute rejection with three IS regimens.

Characteristic	Triple (*n* = 57)	BS (*n* = 241)	SF (*n* = 31)	*P*-value
Acute rejection	3 (5.26)	14 (5.81)	2 (6.45)	0.926
Rejection time				
< 1 month	0 (0.00)	4 (1.66)	1 (3.23)	0.861
2~6 months	2 (3.51)	3 (1.24)	1 (3.23)	
6~12 months	0 (0.00)	2 (0.83)	0 (0.00)	
> 12 months	1 (1.75)	5 (2.07)	0 (0.00)	

### Survival Analysis

#### Overall survival

Till the followed-up end date, 19.15% of the recipients died, and the mortality of triple regimen group was significant higher than BS group (31.58% vs 15.77%, respectively) (*p* = 0.006).

In all recipients, the 1-year, 3-year and 5-year OS rates were 86.40%, 74.02% and 66.14%, respectively. And the 1-year, 3-year and 5-year OS rates were 80.66%, 67.78%, and 63.26% in triple regimen group, 89.25%, 77.88%, and 66.94% in BS group, and 77.18%, 58.81%, and 58.81% in SF group, respectively. No significant difference was observed in three groups for OS rates (*p* = 0.213) (Fig. 2). Of 102 recipients who met Milan criteria, there were 22 (21.57%), 75 (73.53%) and 5 (4.90%) recipients in three groups, respectively.

**Fig 2:** Overall survival rates of recipients in three IS groups (log-rank test, *p* = 0.213).

#### Tumor-free survival

Totally, HCC recurrence was detected in 26.69% (83/311) recipients of all recipients, with a similar proportion of 33.33% (19/57) in triple regimen group, 23.68% (54/228) in BS group and 38.46% (10/26) in SF group (*p* = 0.124).

The 1-year, 3-year and 5-year tumor-free survival rates were 83.45%, 63.87% and 58.09%, respectively. And the 1-year, 3-year and 5-year tumor-free survival rates were 83.90%, 68.08%, and 65.25% in triple regimen group, 84.90%, 64.84%, and 55.73% in BS group, and 70.27%, 43.10%, and 43.10% in SF group, respectively. No significant difference was observed in three groups for tumor-free survival rates (*p* = 0.181) (Fig. 3), either.

**Fig 3:** Tumor-free survival rates of recipients in three IS groups (log-rank test, *p* = 0.181).

#### Graft survival

The 1-year, 3-year and 5-year graft survival rates were 92.13%, 86.09%, and 86.09% in triple regimen group, 92.13%, 89.04%, and 89.04% in BS group, and 88.04%, 88.04%, and 88.04% in SF group, respectively. No significant difference was observed in three groups for graft survival rates (*p* = 0.800) (Fig. 4), either.

**Fig 4:** Graft survival rates of recipients in three IS groups (log-rank test, *p* = 0.800).

Univariate analysis of the risk factors for survival and HCC recurrence was adopted to identify the predictors. Predictors which were significant statistically or certified to be important in previous researches, were included in multivariate analysis. Therefore, the Cox proportional hazard regression multivariate model, which included the following important predictors: IS groups, recipients’ gender, recipients’ age, MELD score, TNM staging, vascular invasion, Milan criteria, preoperative AFP level, number of tumors, diameter of largest tumor and other variables, was conducted. The model showed factors for inferior OS, which were listed as follows: vascular invasion (adjusted HR = 2.015 [1.013, 4.009], *p* = 0.046), preoperative AFP level (>200 ng/ml: adjusted HR = 3.696 [1.340, 10.193], *p* = 0.012; and >400 ng/ml: adjusted HR = 2.372 [1.251, 4.498], *p* = 0.008), and diameter of largest tumor (>5 cm) (adjusted HR = 4.431 [2.086, 9.416], *p*<0.001) (Table 4).

**Table 4:** Cox proportional hazards regression model for overall survival.

Factors^▲^		Reference	Univariate analysis				Multivariate analysis ^☯^			
			HR	95% CI		*P*-value	HR	95% CI		*P*-value
IS groups ^§^										
Group BS	vs.	Triple	0.719	0.408	1.266	0.253	0.486	0.228	1.035	0.061
Group SF			1.348	0.557	3.261	0.508	0.395	0.106	1.468	0.166
Gender ^§^										
Male	vs.	Female	3.522	0.487	25.452	0.212	4.577	0.598	35.033	0.143
Age (years) ^§^										
35~	vs.	18~	0.860	0.116	6.397	0.883	0.562	0.068	4.649	0.593
50~			1.180	0.161	8.626	0.871	1.321	0.168	10.425	0.791
65~			1.552	0.180	13.365	0.689	1.168	0.114	11.961	0.896
Child-Pugh score ^§^										
B	vs.	A	1.050	0.611	1.804	0.860				
C			0.871	0.424	1.790	0.707				
MELD score ^§^										
10~	vs.	6~	0.869	0.508	1.488	0.609	0.658	0.351	1.233	0.191
20~			1.188	0.550	2.564	0.661	1.282	0.534	3.076	0.579
HBV positive ^§^	vs.	No	0.939	0.474	1.861	0.857				
HCV positive ^§^	vs.	No	0.823	0.378	1.790	0.622				
Preoperative diabetes mellitus ^§^	vs.	No	1.167	0.633	2.151	0.620				
Preoperative hypertension ^§^	vs.	No	0.982	0.467	2.066	0.961				
TNM staging ^¶^										
Stage III	vs.	Stage I-II	3.499	1.090	11.229	0.035	1.567	0.421	5.832	0.503
Stage IV			6.932	1.855	25.902	0.004	2.393	0.519	11.028	0.263
Vascular invasion ^§^	vs.	No	4.309	2.570	7.225	<0.001	2.015	1.013	4.009	0.046
Milan criteria ^§^	vs.	No	0.196	0.089	0.431	<0.001	1.236	0.370	4.129	0.731
Preoperative antiviral therapy ^§^	vs.	No	0.744	0.442	1.253	0.267				
Preoperative AFP level, ng/ml ^★^										
200~	vs.	<200	2.391	0.998	5.727	0.050	3.696	1.340	10.193	0.012
400~			2.668	1.576	4.515	<0.001	2.372	1.251	4.498	0.008
Number of tumors ^※^										
Multiple	vs.	Single	1.490	0.859	2.584	0.156	1.467	0.734	2.932	0.278
Diameter of largest tumor, cm ^♦^										
>5	vs.	≤5	5.759	3.307	10.029	<0.001	4.431	2.086	9.416	<0.001

IS: immunosuppression; MELD: model for end-stage liver disease; HBV: hepatitis B virus; HCV: hepatitis C virus; AFP: alpha-fetoprotein; HR, hazard ratio; CI, confidence interval; vs., versus.

^§^ *n* = 329;

^¶^ 7 cases with missing data were excluded;

^★^ 2 cases with missing data were excluded;

^※^ 22 cases with missing data were excluded;

^♦^ 9 cases with missing data were excluded.

^▲^ Adjusted for transplant year in multivariate model.

^☯^ 24 cases with missing data were excluded in multivariate model.

After the multivariate analysis, the association between high HCC recurrence rate and the following factors were also revealed: vascular invasion (adjusted HR = 2.534 [1.369, 4.689], *p* = 0.003), preoperative AFP level (>400 ng/ml) (adjusted HR = 2.878 [1.667, 4.966], *p*<0.001), diameter of largest tumor (>5 cm) (adjusted HR = 4.629 [2.407, 8.901], *p*<0.001) (Table 5).

**Table 5:** Cox proportional hazards regression model for tumor-free survival.

Factors^▲^		Reference	Univariate analysis				Multivariate analysis ^☯^			
			HR	95% CI		*P*-value	HR	95% CI		*P*-value
IS groups ^§^										
Group BS	vs.	Triple	1.057	0.620	1.801	0.838	0.641	0.318	1.295	0.215
Group SF			1.922	0.889	4.155	0.097	1.052	0.370	2.990	0.925
Gender ^§^										
Male	vs.	Female	0.726	0.293	1.799	0.489	1.191	0.398	3.566	0.755
Age (years) ^§^										
35~	vs.	18~	0.439	0.134	1.434	0.173	0.368	0.099	1.362	0.134
50~			0.457	0.141	1.481	0.192	0.653	0.181	2.361	0.516
65~			0.794	0.204	3.086	0.739	0.346	0.069	1.747	0.199
Child-Pugh score ^§^										
B	vs.	A	1.147	0.715	1.841	0.569				
C			0.983	0.530	1.824	0.957				
MELD score ^§^										
10~	vs.	6~	0.998	0.627	1.588	0.993	0.734	0.423	1.274	0.271
20~			1.003	0.476	2.115	0.994	0.995	0.416	2.380	0.991
HBV positive ^§^	vs.	No	1.741	0.801	3.784	0.162				
HCV positive ^§^	vs.	No	0.506	0.219	1.171	0.112				
Preoperative diabetes mellitus ^§^	vs.	No	0.687	0.364	1.298	0.247				
Preoperative hypertension ^§^	vs.	No	0.907	0.468	1.757	0.772				
TNM staging ^¶^										
Stage III	vs.	Stage I-II	4.549	1.429	14.476	0.010	1.325	0.374	4.695	0.663
Stage IV			11.929	3.415	41.677	<0.001	2.609	0.634	10.735	0.184
Vascular invasion ^§^	vs.	No	5.648	3.539	9.013	<0.001	2.534	1.369	4.689	0.003
Milan criteria ^§^	vs.	No	0.123	0.053	0.282	<0.001	1.020	0.324	3.207	0.973
Preoperative antiviral therapy ^§^	vs.	No	1.033	0.633	1.686	0.897				
Preoperative AFP level, ng/ml ^★^										
200~	vs.	<200	1.670	0.659	4.234	0.280	2.139	0.722	6.334	0.170
400~			3.329	2.129	5.205	<0.001	2.878	1.667	4.966	<0.001
Number of tumors ^※^										
Multiple	vs.	Single	2.035	1.225	3.380	0.006	1.776	0.953	3.310	0.071
Diameter of largest tumor, cm ^♦^										
>5	vs.	≤5	6.420	3.969	10.384	<0.001	4.629	2.407	8.901	<0.001

IS: immunosuppression; MELD: model for end-stage liver disease; HBV: hepatitis B virus; HCV: hepatitis C virus; AFP: alpha-fetoprotein; HR, hazard ratio; CI, confidence interval; vs., versus.

^§^ 18 cases with missing data were excluded;

^¶^ 23 cases with missing data were excluded;

^★^ 20 cases with missing data were excluded;

^※^ 38 cases with missing data were excluded;

^♦^ 25 cases with missing data were excluded.

^▲^ Adjusted for transplant year in multivariate model.

^☯^ 40 cases with missing data were excluded in multivariate model.

## Discussion

In recent years, researches of IS therapies developed in transplant recipients were in full swing with conflicting consequences. Many studies agreed that recipients who accepted LTx for HCC were vulnerable by the risk of malignancy especially due to the potential recurrence of the original tumor or the occurrence of de novo tumors. And IS may affect the outcomes in this period [23]. For a long time, evidences indicated that different choices of IS regimens influenced the outcomes of LTx [24], including the survival, HCV recurrence [25, 26] and HCC recurrence [27–29]. For instance, different sirolimus (SRL)-based treatment was relative with survival in HCC, and this was proved by several studies [30–34], although there were some conflicting results among them. Compared with SRL-based treatment, the different treatment of TAC-based was researched rarely, especially for Chinese HCC recipients after LTx. In recent researches the evidence of side effect of steroid based on TAC therapy was found [35], so the steroid-free therapy and induction therapy was applied [36]. However, the effect of these new therapies did not reach an agreement in all researchers [37–39]. In addition, in these studies, the grouping was simple. In this study, the grouping was delicate and the comparison was comprehensive. This may be helpful to explore the truth of different IS therapies based on TAC.

In this study, different therapies based on TAC was evaluated, including the comparison of the IS therapy with and without steroid and the comparison of the induction IS therapy and the standard IS therapy, according to the data of LTx recipients for HCC in China. Most of the clinical characteristics of recipients among three groups were not significant. It indicated that the sample difference preoperative was not remarkable. It was apt to do the next analysis, because this study was a respective study. The similar sample preoperative was easier to obtain real results.

This study also found that the incidence of *De novo* diabetes was comparable among three treatments. Although this result was different from these studies [20, 40], the consistent consequence was obtained in the study [41], which compared the steroid-free IS (daclizumab induction with TAC and MMF) with two standard IS regimens (CS and TAC; CS, TAC and MMF) for LTx recipients with chronic hepatitis C. Besides this study, all of the researches mentioned above demonstrated a trend toward less postoperative diabetes in steroid-free recipients (even the trend was not all statistically significant [41]). Similar to these findings, several studies showed no difference in HBV recurrence [20, 40] and HCC recurrence rate [20] between steroid-based regimens and steroid-free regimen, but higher incidences of biliary complications, graft dysfunction and pleural effusion [20] was observed in SF group. Moreover, several researches reported the negative results of acute rejection rate [20, 41] and rejection time, which were equivalent to this study. All of these findings implied that steroid-free therapy has no clear advantages in comparison with traditional IS therapy in LTx for different etiologies.

Cai et al. [42] found that induced IS improved graft and patient survival for most categories of organ transplants. But in this study, no significant differences were found in the OS rates (*p* = 0.213), tumor-free survival rates (*p* = 0.181) or graft survival rates (*p* = 0.800) among three groups. The experience [43], which was tested in pediatric LTx recipients who were treated with steroid-free and TAC-basiliximab-based IS regimen, compared with TAC-steroid regimen, also confirmed the consequence of patient and graft survivals in this study. Study of Xing *et al*. found that no differences in patients and disease-free survival rates in recipients who received steroid-free (instead of basiliximab) therapy compared with steroid-contained therapy, but a higher disease-free survival rate in recipients who met Milan criteria received basiliximab therapy, compared with steroid therapy [20].

However, there are also some limitations of this study. First, as a retrospective study, the data were irretrievable and limited. Second, steroid-free regimen was applied cautiously for HCC patients, who were advanced TNM stages or some other necessary conditions in this center. Therefore, the small sample size of steroid-free group may impact the results of the comparison. Third, the short follow-up length made it difficult to examine the long-term effect of the three IS regimens. Despite of these limitations, this study was one of the rare researches which compared steroid-free regimen with two traditional standard regimens in LTx recipients, especially in Chinese HCC patients. Due to the insufficient researches and inconsistent consequences, more researches were needed urgently.

## Conclusion

In conclusion, this study found that the incidences of complications which included biliary complications and graft dysfunction were higher in recipients who received steroid-free IS regimen, compared with recipients who received induction-contained regimen. And the incidence of pleural effusion was also higher in SF group than in triple-drug regimen group and BS group. But a trend towards less proportion of *De novo* diabetes was revealed in SF group, in addition. However, no significant differences were observed in overall, tumor-free and graft survival in these three IS groups. Furthermore, the rate of acute rejection and rejection time were comparable in three groups. These findings were consistent with the impact of standard IS regimen and steroid-free IS regimen on LTx recipients with chronic HCV. Thus, these findings suggested that steroid-free IS regimen was safe and effective for LTx recipients for HCC, but no clear advantages were revealed in comparison with standard IS regimen or induction-contained IS regimen.
